# Internet of Things and Edge Computing Model Optimization in Physical Training Status and Countermeasures in College Sports Basketball Optional Course

**DOI:** 10.1155/2021/4295319

**Published:** 2021-12-24

**Authors:** Wengang Chen

**Affiliations:** Department of Physical Education, North Sichuan Medical College, Nanchong, Sichuan 637000, China

## Abstract

In recent years, people have paid special attention to their own health status and paid more and more attention to the cultivation of physical fitness. People of different ages have begun physical exercises. As a compulsory course in university, physical education has played a very positive role in the health of students. In order to promote the common development of basketball activities in many sports academies across the country and improve the educational quality of basketball majors, with a view to cultivating basketball and football talents in line with the culture and social development of the times, this article investigates and evaluates the basketball activities of sports coaches in many sports academies, discusses the pros and cons of high school sports in basketball and other related fields, and provides references and suggestions for improvement in the reform of basketball activities in some sports academies. The results of the study found that based on the Internet of Things and edge computing models, physical training in college sports basketball optional courses has been greatly improved compared with traditional physical training methods. Adding adaptive scheduling to Core 1, priority 1 and 5 was distributed on Core 2∼5. Priority 2 tasks tend to be more balanced.

## 1. Introduction

Modern basketball is the epitome of wisdom and adventure, and it is developing in the direction of “physical combined skills, technical combined intelligence, speed combined with rhythm, high intensity, and high risk.” Its development continues to reflect professionalism. Modern basketball is a global era basketball that is significantly different from original basketball or traditional basketball and has its own distinctive characteristics. We can see from the history of basketball development that it is a modern sports event and a type of global modern sports culture that has gradually matured and developed since the formation of modern society in the 1950s. Basketball has the characteristics of integration, appreciation, commercialization, production, and socialization. The basketball strategy is updated rapidly, and offense and defense are more popular. The athletic ability of basketball players is limited, affected by three factors: personal skills, team, and physical fitness. Natural factors can be considered the key to success. The development of modern basketball game culture makes physical training more and more important in basketball.

Physical training is the process of adapting to the needs of training and competition, improving sports performance, changing the center of gravity, improving physical activity, and developing sports quality under the guidance of interdisciplinary. The content of physical training should be selected according to the needs of special competitions and special training, and suitable reports should be selected from three aspects: body type, physical activity, and athletic quality. Physical exercise is conducive to the growth of human bones and muscles, enhances cardiopulmonary function, improves the functional status of the blood circulation system, respiratory system, and digestive system, is conducive to the growth and development of the human body, improves disease resistance, and enhances the adaptability of organisms. As a hot technology, peak computing has been widely used in the commercial field. The main problem of the current system is the integration of different data and the collaboration between different platforms. Since the data belongs to different systems, a unified data model must be created. Although the function of headsets continues to improve, in order to make the overall performance more efficient, the migration of cloud services based on headset performance capabilities and future sizes is essential.

For the research of basketball physical training, experts at home and abroad have many works. Clemente's purpose is to make a useful synthesis of all the research studies of basketball SSCGS and prove the importance of these games to basketball training. Reviewed studies have shown that in the full game, limited dribbling, coaching encouragement, and the use of smaller formats in continuous training programs may increase heart rate response, blood lactate, and excitement [1]. Grabara compares the changes in spinal curvature between young male basketball players and nontraining controls before and after 2 years. The study included 10 basketball players and 11 untrained men [2]. The Rippstein plurimeter is used to determine the curvature of the anterior and posterior spine. Basketball players and their nontraining peers only differed in the first quantification of lumbar lordosis (*P* < 0.05) [3]. Wan and Shan established a deep learning and optimized ant colony algorithm model for basketball technical and tactical decision-making to solve the optimization problem of actual technical and tactical decision-making. This article uses video image-related algorithms. Get the shot frame settings and shot information of the ball. In this article, by analyzing multiple samples of multishot video, a shot frame detection algorithm is proposed. A mathematical model of the shooting frame is established, which can quickly and accurately locate the shooting frame and determine the penalty frame set [4]. Wang and Gao use machine learning technology to build a basketball feature recognition model. In addition, this research mainly takes the basketball characteristic information in the state of basketball goal as the starting point to compare and analyze the detection methods of target detection in the environment. Realize the construction of dynamic ellipsoid bounding box in the state of motion. In addition, this research designed a controlled experiment to verify the analysis of the research model. The research results show that the model proposed in this paper has a certain effect, which can improve the practical guidance of competition and basketball player training [5]. Tsai et al. proposed a VR-based basketball training system, including an independent VR device and a tablet computer. The system is designed to improve players' ability to understand offensive tactics and enable them to execute these tactics correctly. Evaluate the accuracy of the running path and hesitation time of each tactical step for each participant. The results show that the proposed system is useful for learning complex tactics [6]. Daniele et al. aim to evaluate the workload analysis of basketball practice: (1) the impact of the number of different players on physiological and technical needs; (2) the changes of players' reactions in the game over time; and (3) the relationship between the workload of players and their maturity and training age. Studies have shown that changes in the number of players involved will affect the workload of ball training, and the intensity of ball training varies from game to game. Finally, regardless of the player's maturity and training age, ball training can stimulate enough training stimulation [7]. These studies provide some references for this article, but the relevant research time is too short and the reference is unknown, which makes the article not recognized.

The problems in basketball physical training can be summarized as follows: poor understanding of basketball physical fitness theory, which leads to low efficiency of training behavior or even deviation from the goal. Perhaps it is a major factor in the large gap between Chinese college basketball team and that of European and American college basketball teams. On the basis of previous research studies, from the perspectives of coaches and athletes, I investigate and study the current situation of physical training for basketball teams in Beijing colleges and universities and make suggestions based on the existing problems to provide rules for the physical training of college basketball teams in the future.

The innovations of this article are reflected in the following: (1) the edge computing method of basketball sports training is proposed, and the sports training and the Internet of Things are introduced at the same time; (2) based on the optimization of the Internet of Things model, the research and analysis are carried out, and the current situation and countermeasures of physical exercise in college sports basketball are discussed.

## 2. Physical Training in College Sports Basketball Optional Courses

### 2.1. Edge Computing

Edge computing refers to the use of an open platform that integrates network, computing, storage, and application core capabilities on the side close to the source of things or data and provides the nearest service nearby. Its applications are initiated at the edge, which produces faster network service responses and meets the industry's basic needs in real-time business, application intelligence, security, and privacy protection. Edge computing is between physical entities and industrial connections or at the top of physical entities. And by cloud computing, you can still access the historical data of edge computing.

In the MEC network architecture, the computing, storage, and business service capabilities are submerged to the MEC equipment at the edge of the network. The terminal equipment can offload the business to the network edge nodes for localized processing, thereby satisfying the low latency of the 5G network to a certain extent [8, 9]. In addition, the localized processing of the service can make the service closer to the user itself and the wireless network so as to realize the user's perception and utilization of the network location, network load, and wireless resource utilization rate and effectively improve the user experience [10].

The main difference between the MEC network architecture and the traditional cloud computing network architecture is that the MEC network architecture deploys MEC equipment at the edge of the network close to the user [11]. In the MEC network architecture, as the core part of the network, MEC equipment is mainly used to process services locally at the edge of the network. By utilizing the computing resources and storage resources of MEC equipment, the MEC network architecture can meet the needs of users in 5G networks for low latency, location awareness, and high reliability. In addition, MEC equipment can cache the content processed on it and can actively cache related content from the cloud data center based on the characteristics of surrounding users, thereby further reducing service response delay and improving user experience [12]. The edge calculation method is shown in Figure 1.

The mathematical expression is that the number of interpolation nodes on the original function *f* (*x*) is *n* + *l*:

(1) $$\begin{array}{c} y=a_{1}+a_{1}x+a_{2}x^{2}+a_{3}x^{3}+\cdots +a_{n-1}x^{n-1}. \end{array}$$

The expression of Lagrangian interpolation polynomial can be obtained simultaneously:

(2) $$\begin{array}{c} y=p\left(x\right)\sum_{i=0}^{n}y_{i}\prod_{n}\frac{x-x_{j}}{x_{i}-x_{j}}. \end{array}$$

In the real-time mobile face recognition scenario, the service response delay based on the SD-CFN network architecture can be expressed as follows:

(3) $$\begin{array}{c} S={\left\{\frac{\text{Tsak}}{c}+\text{Wm}\right\}}_{\min}+\frac{\text{Tsak}}{\phi c}+Η. \end{array}$$

The total service delay *T*(TA) can be expressed as follows:

(4) $$\begin{array}{c} T\left(\text{TA}\right)=\left\{\frac{\text{Task}}{c}+\text{wm},\frac{\text{Task}}{c_{2}}+\text{wm},\frac{\text{Task}}{c_{3}}+\text{wm},\ldots ,\frac{\text{Task}}{c_{m}}+\text{wm}\right\}+\phi . \end{array}$$

The solution of the task distribution coefficient *δ*i can be transformed into the solution of the vector TA, which is modeled as the following optimization problem:

(5) $$\begin{array}{c} \sum_{\text{i}=1}^{k}\text{TA}\left(i\right)=\text{Task,}\\ I=\prod_{i=1}\left[{\text{Task}}_{\min},{\text{Task}}_{\max}\right]=\prod_{i=1}\left[0,\text{Task}\right]. \end{array}$$

The total service response delay *t* under no-fault conditions can be expressed as follows:

(6) $$\begin{array}{c} t=\max\left\{\frac{D}{C}+Wl,\frac{D_{c}}{C_{c}}+Wl\right\}. \end{array}$$

Based on the stop-and-equal ARQ protocol, the communication delay between computing nodes vi, vj in the CE-IIoT architecture can be expressed as follows:

(7) $$\begin{array}{c} W=\frac{D}{L}\times \frac{T\left(1+P\right)}{1-P}. \end{array}$$

Then, the time delay *T* for the successful transmission of a data packet is calculated as follows:

(8) $$\begin{array}{c} T=\frac{L}{R},\\ W_{vi,vj}=\frac{D}{r}\times \frac{1-l}{1+l}. \end{array}$$

Similarly, the communication delay between MEC device vj and cloud server C can be calculated as follows:

(9) $$\begin{array}{c} W_{\text{c}}=\phi \frac{D}{r}\times \frac{1-P}{1+P}. \end{array}$$

The relationship between the new individual and the original individual is expressed as follows:

(10) $$\begin{array}{c} X_{1}=\lambda X_{1}+\left(1-\lambda \right)X_{2},\\ X_{2}=\lambda X_{2}+\left(1-\lambda \right)X_{1},\\ x=x_{il}+\left(d-x_{il}\right)\left(1-q^{\left(1-g/G\right)\phi }\right), \end{array}$$

where *q* is a random number uniformly distributed in the range of [0, 1], *g* is the current evolutionary algebra, and *G* represents the largest evolutionary algebra.

### 2.2. Physical Training

Human physical fitness is the world's number one sports event and the foundation of sports [13, 14]. Physical training in basketball is indispensable. The methods of physical training in basketball are rich and diverse. Different individual events in basketball have different requirements and focus on physical training [15]. To have a strong physique, exercise is the best method, but blind exercise not only fails to produce results, but may cause injury, so physical exercise must master the correct method to achieve the purpose of physical exercise. The exercise methods include repetitive exercise. This article combines its own practical experience and extracts some methods and methods that are relatively in line with energy metabolism and project characteristics from the many physical training methods and methods of basketball events for experimental research. In addition, from the release of basketball cross-sports and cross-border selection policies and the development trend of basketball, it shows that physical training plays an increasingly important role in basketball training. How to formulate a reasonable basketball physical training plan to improve basketball specific skills, therefore, improving the level of basketball competition, has become a major difficulty in basketball training [16, 17]. Among them, the invention of basketball is also very interesting. Basketball was invented by the American James Naismith in 1891. At that time, he was teaching at the YMCA International Training School in Springfield, MA, USA. Because the local area is rich in peaches, the children here also like to play the game of throwing the ball into the peach basket. This inspired him to create basketball games based on the characteristics of football, hockey, and other ball games.

### 2.3. Internet of Things

The Internet of Things is no different from the current cloud computing technology and wireless communication technology. These technologies can be applied to almost any product [18, 19]. The Internet of Things can determine the precise balance of products and services, as well as the corresponding personal health and other aspects [20, 21]. The Internet of Things is the oldest company in the world and has become the leading authority for the entire company. The essence of the Internet of Things is the Internet, but it also has many characteristics of its own. The Internet is a type of information transmission, and this process always applies to the same provider. In the real network process, many real-time interactions are known, that is, communication and information exchange between objects and people [22]. The actual characteristics of the Internet of Things are important in the following aspects:

1. *Internet Characteristics*. The Internet of Things is a new type of network, and the entire solution is also the communication between things and things and between people and things. Although the current form is different, the Internet of Things is also the Internet technology in the real world. Therefore, the development of its core technology the foundation is also Internet technology [23]. The basic laws and characteristics of the Internet of Things from the perspective of communication objects and processes; the information interaction between things and between people and things is the core of the Internet of Things. The basic laws and characteristics of the Internet of Things can be summarized as overall perception, reliable transmission, and intelligent processing.
2. *Understand the Characteristics*. The Internet of Things can achieve a certain degree of self-control and a consistent understanding of design. The Internet of Things can finally effectively analyze and process large amounts of data, mainly using cloud computing technology for decision-making and management [24]. The architecture of the Internet of Things is shown in Figure 2.

Using the zero-forcing algorithm to estimate *H*_*B*_, we get

(11) $$\begin{array}{c} H_{AB}=\frac{x_{A}^{T}}{x_{A}},\\ y_{B}=H_{0}+\frac{x_{A}}{{\left\|x\right\|}^{2}}n_{b}. \end{array}$$

Among them, (•)^*T*^ represents the transposition of a vector or matrix, and ‖*x*‖ represents the modulus of the vector *x*_*A* _.

With the development of basketball, the antagonism of the game is getting stronger and stronger. Modern basketball is developing in the direction of strong confrontation, fast-paced, high-speed, high-skill, and high-altitude combat. And this development trend requires good physical fitness and technology as a guarantee. Basketball is a competitive sport, which follows the four elements of competitive ability: technology is the foundation, tactics are the means, the body is the guarantee, and the psychology is the fundamental. Only with superb basketball skills can you gallop on the court, and at the same time, with sophisticated tactics, you can move forward and retreat more than once on the court. Healthy physical fitness is an important guarantee for playing well in every game, and good psychological quality is also the essential essence of being a basketball player. Among the four elements, the body is the guarantee for everything. If an athlete does not have good physical fitness, then all techniques and tactics are empty talk. The body needs physical energy as support, and only through scientific and systematic physical training can the athletes' bodies be exercised to a level that meets the specific characteristics of basketball. Bob sends *x*_*B*_ with a power of PB; then,

(12) $$\begin{array}{c} h_{BA}=\kappa \left(\chi +\frac{\phi }{T}\right),\\ h_{E}=\phi \pi \left(\chi +\frac{\phi }{T_{B}}\right). \end{array}$$

Therefore, the key capacity *C*_*S*_ that can generate the key is

(13) $$\begin{array}{c} C_{S}=\max I\left(y_{A};y_{B}\right). \end{array}$$

General physical fitness includes endurance, speed, strength, agility, flexibility, and coordination. Endurance is one of the important indicators of athletes' physical fitness. There are many sports such as ball games, cycling, swimming, mountaineering, and track and field middle- and long-distance running, race walking. The improvement of technical level and the achievement of competition results often depend on the level of endurance. And some sports that do not require high aerobic endurance, such as weightlifting, diving, and gymnastics, also have higher requirements for specific endurance. Good endurance is also an important prerequisite for accelerating body recovery after heavy training. Endurance quality can be divided into many types according to different standards. For different types of endurance, different training methods should be used during training. It can be seen that the following Markov relationship is established:

(14) $$\begin{array}{c} h_{BA}⟷y_{A}⟷h_{0}⟷y_{B}⟷h_{AB}. \end{array}$$

According to the Markov relationship:

(15) $$\begin{array}{c} I\left(y_{A};y_{B}\right)\leq I\left(h_{BA};h_{AB}\right). \end{array}$$

In the definition of Markovian nature, “now” refers to a fixed moment, but in practical problems, it is often necessary to generalize the concept of “now” in Markovian nature to stop time (see random process). For example, to investigate the Brownian motion on a plane starting from the center of a circle, if we want to study the conditional independence of events before and after the moment *T* when it first reaches the circle, here *T* is the stop time, and *T* is considered “now.”

## 3. Internet of Things and Edge Computing Model Optimization in the Physical Training Status and Countermeasures of the College Sports Basketball Elective Course Analysis of Experimental Results

### 3.1. Research and Analysis of IoT Model Optimization

In the embedded multicore SoC convergence node, if the task buffer capacity is full, blocking will occur when the next task arrives and the execution core at this time has not completed the task being executed. Therefore, the blocking probability can be approximately equivalent to the probability that the node cache is full [25, 26].

The relationship between the probability that the node cache is full and the task cache capacity is shown in Figure 3. As the task cache capacity increases, the probability of each execution core task cache being full begins to decrease rapidly, and when the task cache capacity exceeds 4, the decrease speed begins to slow down. When task cache capacity 8 is reached, increase the task cache capacity. The probability of Core 1 and Core 2's cache being full does not change very much; the probability of Core 3's cache being full is lower than 0.2, while the probability of Core 4 and Core 5 being full is gradually approaching zero.

Integrating the relationship curve between the utilization rate of each execution core of the embedded multicore aggregation node and the task cache capacity and the relationship curve between the cache full probability and the task cache capacity, the selected task delay capacity is called the task cache capacity. In this way, under the limited consumption of hardware cache resources, the utilization of each execution core of the embedded multicore can be maximized, and the degree of congestion of the system can be effectively alleviated.

According to the performance evaluation of embedded multicore SoC queuing network molding, the arrival rate of different priority tasks of each execution core is obtained. Since the hardware resources occupied by Core 2∼5 are basically the same, their task processing capabilities are basically the same. If the load of each core differs greatly, the processing capabilities of the entire system will not be high, so effective task adaptation scheduling methods are required.  Figure 4 shows the distribution of the arrival rate of each execution core before and after the adaptive scheduling conversion method is used in the actual test. It can be seen that after adding adaptive scheduling to Core 1, the tasks of priority 1 and priority 2 distributed on Core 2∼5 tend to be more balanced.

Among them, the size of the change rate of the node position of the perception layer of the Internet of Things determines the speed of the change of the topology of the perception layer of the Internet of Things, which is a direct reflection of the stability of the perception layer of the Internet of Things [27, 28]. In the simulation process of this article, the change rate of the moving position of the sensing layer node of the Internet of Things is set from 0 m/s to 35 m/s, with an increment of 5 m/s each time. In this process of gradual change, the performance of the gateway access-oriented routing protocols GARP and ODTM protocols proposed in this paper have declined to varying degrees.

The comparison of the average end-to-end delay between the gateway and the source node at different rates of node location changes is shown in Figure 5(a). As the rate of node location changes increases, the routing facing gateway access the average end-to-end delay between the gateway and the source node of the GARP and ODTM protocols has increased to varying degrees. This is because as the rate of node location changes increases, the network topology changes more drastically, resulting in frequent links the disconnection fails, which increases the number of restarts of the route discovery process, which increases the average end-to-end delay between the gateway and the source node. Among them, the comparison of the packet delivery rate between the gateway and the source node at different rates of node location changes is shown in Figure 5(b). As the rate of node location changes increases, the gateway access-oriented routing protocol GARP. The packet delivery rate between the gateway and the source node of the ODTM protocol is decreasing. This is because the increase in the rate of node location changes has caused the previously established link to continue to fail, and the packet loss phenomenon is becoming more and more serious. However, in the same scenario, the packet loss of the gateway-oriented routing protocol GARP is slightly less. This is because the clustering and cluster head election algorithms optimized for gateway selection consider the energy problem of nodes, and the selected cluster head nodes will not have less remaining energy. Data packets are transmitted between cluster head nodes with higher energy, which reduces the situation that cluster head nodes discard packets due to low energy.

In the multigateway multipath transmission method, when the load is light, the average end-to-end delay between the gateway and the source node is higher than the previous two cases, mainly because a certain number of gateways need to be selected from the candidate cluster heads, so that increases the routing delay. However, the benefits of this method are gradually reflected when the number of connections increases and the load on the network becomes heavier. This method means that the optimized cluster and cluster head election algorithm selected by the gateway takes into account the energy problem of the node, and the selected cluster head node will not have less remaining energy. At this time, the number and quality of gateways are both effective and reasonable due to the multigateway and multipath transmission method. The average end-to-end delay between source nodes is lower than adding the previous two cases because the performance of the path selected by this method is more superior, and the load balance is better than the previous two.

Figure 6(a) shows the packet delivery rate between the gateway and the source node in three different situations. It can be seen from the figure that the packet delivery rate between the gateway and the source node decreases with the continuous increase of the number of connections in the three different cases, but the magnitude of the decrease is different. The packet delivery rate between the gateway and the source node is the lowest in the single-path transmission method using only one gateway. In Figure 6(b), we can see how the parameter of the network overhead during the transmission between the gateway and the source node changes with the number of connections in the above three cases. It can be seen from the figure that the network overhead of the three methods of gateway and source node transmission decreases with the continuous increase of the number of connections, but the multipath transmission method and the multigateway multipath are simply used by one gateway. When the gateway and source node of the transmission method transmit, the network overhead tends to decrease with the increase of the number of network connections.

### 3.2. Status Quo and Countermeasures of Physical Training in College Sports Basketball Elective Courses

Table 1 shows that 54.9% of students love and love basketball very much. 83.2% of the students are very interested and interested in the basketball elective course, and 43.1% of the students prefer the basketball elective course. It can be seen that students like basketball and choose coaching activities according to their needs. However, many students do not like basketball activities, which shows that they love basketball but do not like basketball activities. Just like they are more enthusiastic about NBA games, they like more ornamental basketball games, but they are not very keen on basketball activities, and some students like to devote themselves to the game and look forward to the fullness of the game.

It can be seen from Table 2 that 95.1% of the students' initial training motivation is to obtain credits, 56.2% are to improve their basketball skills, and 49.1%, 28, 1%, and 28.1% are exercises, physical conditions, and social needs per game.

Basketball chess training is a course with basic skills as the main content. The teaching content of basketball practice is shown in Table 3. 43.9% of students reported the content of technical and process analysis. The proportions of drinking and accumulating habits in basketball are relatively small, at 13.9% and 8.1%, respectively. In practice, basic technical content accounted for 99.5% and core training content accounted for 29.3%, while the shares of basketball and basketball games are 22.9% and 25.2%, respectively. There are few plans for these two training contents.

The so-called “training for a thousand days, using the soldiers for a while,” without the boring training of the week, is the glory of the game. It can be seen from Table 4 that there is a sharp contrast between the coaches and the athletes' data. In the basketball team's special physical training, only 39% of the athletes think it is necessary to increase the training methods and time of the special physical training, while most of the athletes believe that it is unnecessary. Obviously, basketball players have insufficient knowledge and understanding of specific physical training. The main reasons are as follows: athletes' attitude towards specific physical training is too negative; athletes' time and energy cannot be devoted to specific physical training; and the boringness of specific physical training cannot stimulate athletes' interest.

The basketball game in the twenty-first century is a confrontation between players in time and space. In a basketball game, every pass and every shot has extremely high requirements for upper limb strength, especially in the case of fierce confrontation, stalemate, excessive physical exertion, psychological and physical changes, the effect is particularly effective protrude. In basketball games, passing, layups, and shooting are not only dependent on the strength of the arm, but also rely on the strength of the fingers and wrist to control the rotation, height, strength, and stability of the ball. It can be seen that the strength of the upper limbs is particularly important in the basketball game.

It can be seen from Figure 7 that the common training methods used by the basketball team in upper limb training, the number of training groups, and the number of training are also different, the push-up training is self-determined according to the strength of the athletes themselves, and the requirements for the athletes are relatively low.

The lower limb strength training of basketball players is based on explosive power and special strength as the core. The lower limb training mainly improves athletes' physical confrontation, breakthrough, start-up, rapid change of direction, continuous jumping, steals, etc., which have obvious effects. Many athletes' knee injuries of varying degrees are closely related to the seriousness of the usual strength training and the methods of training.

In the basketball team, athletes have poor physical fitness, lack of physical fitness, weak lower limb strength, and no instantaneous explosive power. It can be seen from Figure 8 that most coaches of the basketball team pay more attention to explosive training but ignore the strength training of the knee joint, which shows that coaches do not pay enough attention to health care and injury prevention training in sports training.

## 4. Discussion

The future 5G network needs to support a large number of rich applications. Because MEC has the above advantages, in the 5G network, the application scenarios of MEC mainly focus on the generation and processing of local data so as to meet the requirements of different services for low latency and high bandwidth. The industrial Internet of Things is one of the key technologies to realize the digital transformation of the industrial field. The relevant production data in the Industrial Internet of Things is generated locally, and most of these data need to be processed in real time. Uploading the data to the cloud for processing will face unbearable time delay. At the same time, industrial IoT data can only be transmitted locally in a closed loop due to security requirements. The MEC technical solution satisfies the abovementioned requirements in the industrial Internet of Things. In the MEC-based industrial Internet of Things, industrial production equipment, smart robots, smart terminals, sensors, etc., can upload production data, status, and other information during the production process to MEC equipment for real-time processing so as to obtain an efficient production plan and complete the coordination of different links, which improves production efficiency.

Although the attributes of edge devices continue to improve, in order to make the overall performance more efficient, the migration of cloud services based on edge computing performance capabilities and future dimensions is indispensable. In recent years, society has increasingly entered the “big data” era, and the emergence of cloud computing has increased the demand for big data and application capabilities. Whether it is cloud, fog, or edge computing, it is only a method or mode for realizing the computing technology required by the Internet of Things and smart manufacturing. Strictly speaking, there is no essential difference between fog computing and edge computing. Both are calculations provided close to the field application. In its essence, they are all relative to cloud computing. However, due to its high application requirements, this computer architecture cannot be promoted during its use. How to use existing resources for data collection has become a prerequisite for restricting the development of big data services. Special physical training is a complicated process. In a sense, it requires professional training with a variety of personal advantages according to the characteristics of age and gender.

Mobile users can utilize the higher resources of the server by transferring computing tasks to the MEC server. Emerging and more mobile applications will benefit from MEC by moving their intensive functions from MEC servers to cloud computing. For edge laptop users, we assume that all tasks required for computing are independent of each other. On this basis, a new perspective of the transfer process is given; that is, it is not decided whether to proceed alone. Delete the task, but authorized to perform the task. On this basis, by writing a load model that combines the two factors of containment and power consumption, the optimization problem of load reduction is proposed. Subsequently, the low-time complexity binary particle swarm optimization algorithm and the Johnson algorithm in the dual-engine design are used to optimize the problem. Finally, the algorithm was verified by simulation tests, and the performance was compared with other algorithms. Regarding the binary particle swarm optimization algorithm, the particle swarm optimization algorithm is an algorithm for solving continuous space problems. However, if you want to apply it to the feature selection problem to find the necessary 0/1 strings, some minor modifications have to be made to solve the discrete space problem. Of course, one of the simplest methods is to set a threshold value for the position value. If the threshold value is exceeded, set it to 1, otherwise it is set to 0, so that the *N*-dimensional position vector of the continuous space is converted into the 0/1 string of the discrete space. However, it does not make sense to explain this, so the binary particle swarm optimization algorithm appeared. Its improvement to the particle swarm optimization algorithm is as follows: the speed formula remains unchanged, a sigmoid function is added, and the position formula is redefined.

## 5. Conclusion

Although students' practical ability can be exercised and improved by participating in certain social practice activities, most of the improvement of students' professional ability is through the accumulated training effects of practical classes in the school. Basketball professional courses include both professional basic courses, basketball theory courses and practical courses. Therefore, all factors that can affect professional basic courses, basketball theory courses and practical courses will affect basketball professional courses. Among these influencing factors are teachers and students. The relationship and communication status are an important factor that needs to be paid attention to by all parties. In the teaching, the phenomenon of “emphasizing knowledge accumulation, neglecting knowledge application,” “emphasizing theory instillation, neglecting practical teaching operation” is common; in professional course teaching, “emphasizing professional knowledge, neglecting compound knowledge” and “less forward-looking courses, less reflecting on physical education,” “new achievements in the field.” The teaching method is relatively traditional, and the teaching method is single. Sports colleges should closely integrate the actual needs of the society for talents in the training goals of sports training. They can start to train some outstanding basketball students to the direction of basketball trainers and physical fitness teachers to meet the diverse development needs of modern basketball. The main research direction of this article is based on the Internet of Things and edge computing models to explore the optimization status and countermeasures of sports basketball training courses in colleges and universities. It conducts an investigation and research on sports basketball training courses in colleges and universities. However, due to the limitations of experimental techniques, the number of samples investigated is not very large, and there are certain errors. We will further explore them in the follow-up.

## Figures and Tables

**Figure 1:** Edge computing method.

**Figure 2:** IoT architecture.

**Figure 3:** The relationship between the probability that the cache is full and the capacity of the task cache.

**Figure 4:** Comparison of task reach rate before and after adaptive scheduling.

**Figure 5:** Comparison of average end-to-end delay between gateway and source node and comparison of packet delivery rate.

**Figure 6:** Comparison between gateway and source node.

**Figure 7:** Basketball team special physical capacity training one upper limb.

**Figure 8:** Basketball team's special physical capacity training of lower limbs.

**Table 1:** Survey results of students' interest in basketball optional courses and their likes.

Interest in basketball	Frequency	Percentage	Like degree of basketball option class	Frequency	Percentage
Very interested	559	33	Like very much	388	21.3
Interested	893	50.2	Like	569	33.6
Generally	198	9.8	Generally	451	23.2
Not interested in	71	4.6	Do not like	309	18.9
Dislike	26	2.4	Do not like it very much	32	2

**Table 2:** Survey results of students' motivation to study basketball optional courses.

Options	Frequency	Percentage	Options	Frequency	Percentage
Strengthen the system	491	28.1	Self-fulfillment	228	12.8
Improve basketball	978	56.2	Gain academic credit	1802	95.1
Lay the foundation for lifelong exercise	339	20.3	Admire the teacher	152	8.8
Social needs	459	25.9	Entertaining body and mind	861	49.1

**Table 3:** List of teaching contents of basketball optional course.

	Options	Frequency	Percentage		Options	Frequency	Percentage
Theoretical part	Basketball overview	141	8.1	Practice part	Basketball game	429	25.2
	Rules and judgments	38	2.1		Basic technique	1761	99.5
	Tactical analysis	781	43.9		Basic tactics	497	29.3
	Injury and health knowledge	251	13.9		Basketball game	101	22.9

**Table 4:** Analysis of the level of awareness of athletes on specific physical fitness.

	It is necessary	Percentage	No need	Percentage	Unclear	Percentage
Equipped with a full-time physical coach	81	93	6	7	0	—
Strengthen special physical training	60	71	19	31	3	6
Increase training time for specific physical fitness	40	39	40	50	11	13

## Data Availability

No data were used to support this study.
